RETRACTED

# Clinical Efficacy of Budesonide/Glycopyrronium Bromide/Formoterol in the Treatment of Patients with Acute Respiratory Distress Syndrome and Its Effect on Inflammatory Factors

**DOI:** 10.1155/2022/8150444

**Published:** 2022-04-28

**Authors:** Haiying Liu, Zhengyan Wang, Lijun Ren, Guiqin Zhang, Dan Zhao, Yanli Guo, Lijuan Wang, Hong Feng

**Affiliations:** ^1^Department of Respiratory and Critical Care Medicine, The Fourth Hospital of Baotou, Baotou City, Inner Mongolia, China; ^2^Endoscopy Center, The Fourth Hospital of Baotou, Baotou City, Inner Mongolia, China; ^3^Department of Infectious Diseases, Baogang Third Hospital of Hongci Group, Baotou City, Inner Mongolia, China; ^4^Department of Respiratory and Critical Care Medicine, Hohhot First Hospital, Hohhot, Inner Mongolia, China; ^5^Department of Nursing, The Fourth Hospital of Baotou, Baotou City, Inner Mongolia, China; ^6^Department of Nephrology and Hematology, The Fourth Hospital of Baotou, Baotou City, Inner Mongolia, China; ^7^Medical Department, The Fourth Hospital of Baotou, Baotou City, Inner Mongolia, China

## Abstract

**Objective:**

To examine the clinical efficacy of budesonide/glycopyrronium bromide/formoterol (Breztri Aerosphere) as an adjunct to acute respiratory distress syndrome (ARDS).

**Methods:**

A prospective study enrolled 120 patients with pulmonary endogenous ARDS admitted to the Department of Critical Care Medicine at the Fourth Hospital of Baotou from January 2017 to January 2020, and all enrollments were assigned (1 : 1) to receive conventional treatment (control group) or Breztri Aerosphere (study group).

**Results:**

Breztri Aerosphere was associated with a significantly higher total efficacy versus conventional treatment. Breztri Aerosphere resulted in significantly lower acute physiology and chronic health evaluation scoring system (APACHE II) scores and Murray lung injury scores versus conventional treatment. Both groups saw an increase in the partial pressure of carbon dioxide (PCO2), partial pressure of oxygen (PO2), and oxygen saturation (SaO2) after treatment, with higher levels seen in patients given Breztri Aerosphere. After treatment, systemic vascular resistance (SVR) in both groups rose markedly, with greater elevation witnessed in the study group. The patients given Breztri Aerosphere showed significantly lower levels of pulmonary vascular resistance (PVR), mean pulmonary arterial pressure (MAPA), pulmonary artery wedge pressure (PAWP), interleukin-6 (IL-6), interleukin-10 (IL-10), tumor necrosis factor-alpha (TNF-*α*), and procalcitonin (PCT) versus those receiving conventional treatment. The patients experienced shorter mechanical ventilation time and intensive care unit (ICU) time after treatment of Breztri Aerosphere versus conventional treatment.

RETRACTED

**Conclusion:**

Adjuvant therapy with Breztri Aerosphere in ARDS can significantly lower APACHE II scores and Murray lung injury scores, improve blood gas indexes and pulmonary circulation function indexes, and shorten mechanical ventilation time and ICU time, which may be attributed to its improvement of organism inflammation status and reduction of inflammatory factors.

## 1. Introduction

Acute respiratory distress syndrome (ARDS) is an acute diffuse lung injury characterized by alveolar capillary endothelial and alveolar epithelial cell injury, which is characterized by acute onset, respiratory distress, and hypoxemia. The clinical outcomes after conventional oxygen therapy are modest, and the pathogenesis of the disease remains elusive [1, 2]. ARDS manifests as lung edema due to inflammatory alveolar exudate and increased pulmonary vascular permeability, which results in disturbed gas exchange and acute deterioration [3]. Invasive mechanical ventilation is a common treatment method for patients with ARDS but is associated with certain lung injuries [4]. TCM believes that qi deficiency and blood stasis are the basic pathogenesis of gastrointestinal dysfunction in ARDS patients treated with mechanical ventilation. Effective pharmacotherapy can be crucial in the treatment and prognosis of ARDS to enhance survival and shorten mechanical ventilation time [5]. Breztri Aerosphere, composed of budesonide/glycopyrronium bromide/formoterol, is a triple combination of the glucocorticoid budesonide, the long-acting *β*2 agonist formoterol fumarate, and the long-acting cholinergic receptor antagonist glycopyrronium bromide [6]. The combination of the three drugs with different mechanisms of action potentiates their efficacy, with well-recognized efficacy in the treatment of chronic obstructive pulmonary disease (COPD); however, the efficacy of the drug for ARDS is poorly understood. Accordingly, budesonide/glycopyrronium bromide/formoterol (Breztri Aerosphere) was applied in 120 cases of ARDS admitted to the Department of Critical Care Medicine at the Fourth Hospital of Baotou from January 2017 to January 2020. The report is discussed in this study.

## 2. Materials and Methods

### 2.1. General Information

A prospective study enrolled 120 patients with pulmonary endogenous ARDS admitted to the Department of Critical Care Medicine at the Fourth Hospital of Baotou from January 2017 to January 2020, and all enrollments were randomized (1 : 1) into a control group and a study group. This study was conducted in accordance with the Declaration of Helsinki [7] and was reviewed by the Ethics Committee of the Fourth Hospital of our hospital.

RETRACTED

### 2.2. Inclusion and Exclusion Criteria

#### 2.2.1. Inclusion Criteria

The inclusion criteria were as follows: (1) patients aged 18 to 65 years; (2) patients met the Berlin diagnostic criteria for ARDS [8]; (3) patients were diagnosed with ARDS within 1 week and were treated with mechanical ventilation for <24 hours; (4) patients could understand the purpose and risks of the study; and (5) patients provided written informed consent.

#### 2.2.2. Exclusion Criteria

The exclusion criteria were as follows: (1) patients with a diagnosis of ARDS for more than 1 week; (2) during pregnancy, lactation, or perinatal period; (3) with severe terminal stage lung diseases, malignancies, or other clinically relevant diseases that affect the study outcome; (4) with a predicted risk of death >80% within 24 h; (5) with ECMO or mechanical ventilation; and (6) patients who were unwilling or unable to follow the study protocol.

### 2.3. Treatment Methods

#### 2.3.1. Treatment for the Control Group

The control group was given conventional treatment, including etiological treatment, fluid management, sedation and analgesia, and nutritional support. Invasive mechanical ventilation was provided if necessary. (1) Etiological treatment: the etiology of ARDS involves various fields such as trauma, infection, and burns, and aggressive and effective etiological treatment is the key to the treatment of ARDS. Timely hemostasis and surgery were provided for trauma-induced ARDS, and patients with sepsis-related ARDS received early fluid resuscitation, anti-infective treatment, and vasoactive drugs. (2) Fluid management: fluid intake was limited on the basis of efficient organ perfusion, with a reasonable balance between the use of crystalloid and colloid fluids, and diuretics were given appropriately, with the hemodynamics of the patients being closely monitored. (3) Sedation and analgesia: appropriate sedation and analgesia were administered to relieve the patient's stress state and improve the coordination between the body and the ventilation machine. A sedative goal of a Ramsay sedation score of 3–4 was established for the patients if their condition allowed, and they were awakened daily to ensure intermittent wakefulness. (4) Nutritional support: given the rapid metabolism of ARDS patients, timely and proper enteral nutrition support was given on the premise of normal intestinal function.

#### 2.3.2. Treatment for the Study Group

On the basis of the control group, the study group was given budesonide/glycopyrronium bromide/formoterol (Breztri Aerosphere) (manufacturer: AstraZeneca Dunkerque Production, France, NMPA Approval No. H20190063, size: 120 snap/172 *μ*g, ingredients: budesonide 160 *μ*g, glycopyrronium bromide 7.2 *μ*g, and formoterol fumarate 4.8 *μ*g) as adjunctive therapy, 2 inhalations per dose, twice daily, administered only by transoral inhalation. The clinical efficacy of all patients was evaluated after 10 consecutive days of treatment.

RETRACTED

### 2.4. Observational Indicators

#### 2.4.1. Clinical Efficacy

Clinical efficacy was classified as cured, effective, and ineffective based on the patients' clinical symptoms, blood gas, and imaging. Cured: the dyspnea disappeared, the blood gas indices returned to a normal level, and the imaging showed the dissipation of lung shadows or only thickening of lung texture. Effective: respiratory distress was reduced, blood gas indices were improved, and imaging showed good absorption of lung shadows. Ineffective: the symptoms of the patients did not meet the abovementioned criteria. Total efficacy = (the number of cured patients + the number of effective patients)/the total number of patients^*∗*^100%.

#### 2.4.2. Acute Physiology and Chronic Health Evaluation Scoring System (APACHE II) Scores and Murray Lung Injury Scores

Before and after treatment, patients' APACHE II scores [9] and Murray lung injury scores [10] were recorded. The APACHE II scores include three domains of acute physiological score (12 physiological indicators), age score, and chronic health score. The higher the score, the more severe the disease and the worse the prognosis. Murray lung injury scores include four domains of X-ray score, hypoxemia score, positive end-expiratory pressure score, and lung compliance score, with the total score = the sum of the scores for each parameter/the sum of the number of parameters used. A higher Murray lung injury score indicates more severe lung injury, where 0.25–0.5 is classified as mild to moderate lung injury and >2.5 is classified as severe lung injury.

#### 2.4.3. Blood Gas Analysis

In both groups, radial artery blood was collected for arterial blood gas monitoring before and after 5 days of treatment to determine the partial pressure of carbon dioxide (PCO_2_), partial pressure of oxygen (PO_2_), and oxygen saturation (SaO_2_).

#### 2.4.4. Pulmonary Circulation Function Indexes

Systemic vascular resistance (SVR), pulmonary vascular resistance (PVR), mean pulmonary arterial pressure (MAPA), and pulmonary artery wedge pressure (PAWP) were recorded by cardiac ultrasound and the PiCCO monitor.

#### 2.4.5. Changes in Inflammatory Factors

Fasting venous blood was collected from patients on the day after admission and after 10 days of treatment, and peripheral blood interleukin 6 (IL-6), peripheral blood interleukin 10 (IL-10), tumor necrosis factor-alpha (TNF-*α*), and procalcitonin (PCT) were determined by an enzyme-linked immunosorbent assay (ELISA).

RETRACTED

#### 2.4.6. Survival Curve

All patients were followed up for 28 days. The survival rate was analyzed by the Kaplan–Meier test, and the survival curve was obtained.

### 2.5. Statistical Analyses

SPSS 22.0 software was used to organize and statistically analyze the data, and GraphPad Prism software was used to plot the graphics. The measurement data were expressed as mean ± standard deviation/±s. The *t*-test for two independent samples was used for comparison between groups, and the *t*-test for paired samples was used for comparison within a group. Count data were expressed as rates (cases (*n*%)), and the chi-square test was used to verify the presence or absence of statistical differences. Kaplan–Meier curves were used to plot survival curves. The difference was considered statistically significant with *α* = 0.05 as the threshold of significance.

## 3. Results

### 3.1. Comparison of General Information

In the control group, age was 62.35 ± 12.23 years, the gender ratio of male/female was 38/22, and the BMI was 26.45 ± 5.31 kg/m^2^. In the study group, age was 60.46 ± 14.35 years old, the gender ratio of male/female was 41/19, and the BMI was 25.97 ± 6.43 kg/m^2^. As shown in Table 1, the two groups showed comparable general information such as age, gender, BMI, and underlying diseases (*P* < 0.05).

### 3.2. Comparison of Clinical Efficacy

Results in Table 2 show that the control group had 12 cases of cured, 34 cases of effective, and 14 cases of ineffective, with a total efficacy of 76.67% (46/60). The study group had 16 cases of cured, 38 cases of effective, and 6 cases of ineffective, with a total efficacy of 93.33% (54/60). Breztri Aerosphere was associated with a significantly higher total efficacy versus conventional treatment (*χ*2 = 6.539, *P*=0.011).

### 3.3. Comparison of APACHE II Scores and Murray Lung Injury Scores

Results in Figure 1 present no great disparity in the APACHE-II scores and Murray lung injury scores between the two groups before treatment (*P* > 0.05). Breztri Aerosphere resulted in significantly lower APACHE II scores and Murray lung injury scores versus conventional treatment. (*P* < 0.05).

### 3.4. Comparison of Blood Gas Indexes

Before treatment, the two groups showed similar results in blood gas indexes including PCO_2_, PO_2_, and SaO_2_. After treatment, the three levels of index were all elevated in both groups, with higher results seen in patients given Breztri Aerosphere (*P* < 0.05) (Table 3).

### 3.5. Comparison of Pulmonary Circulation Function Indexes

Results in Figure 2 demonstrate no significant difference in SVR, PVR, MAPA, and PAWP between the two groups before treatment (*P* > 0.05). After treatment, SVR in both groups rose markedly, with greater elevation witnessed in the study group (*P* < 0.05).

RETRACTED

### 3.6. Comparison of Inflammatory Factors

Before treatment, the two groups showed no significant difference in the levels of IL-6, IL-10, and PCT (*P* > 0.05). The patients given Breztri Aerosphere showed significantly lower levels of PVR, MAPA, PAWP, IL-6, IL-10, TNF-*α*, and PCT versus those receiving conventional treatment (*P* < 0.05) (Figure 3).

### 3.7. Comparison of Mechanical Ventilation Time and ICU Time

In Table 4, mechanical ventilation was applied for 52 patients in the control group with unsatisfactory efficacy after drug therapy, while the study group had 49 cases. No significant difference was detected in the proportion of patients receiving mechanical ventilation (*P* > 0.05). The patients experienced shorter mechanical ventilation time and ICU time after treatment of Breztri Aerosphere versus conventional treatment (*P* < 0.05).

### 3.8. Comparison of the Survival Curve

Results in Figure 4 reveal that within 18 days after admission, 5 cases of death were reported in the control group, with a death rate of 8.33%, and 2 cases of death were reported in the study group, with a death rate of 3.33%, where no significant difference was seen between the two groups (*P* > 0.05). The two groups also did not differ in their survival curves (*P* > 0.05).

## 4. Discussion

ARDS is a noncardiogenic pulmonary edema and a diffuse pulmonary inflammatory syndrome [11], with rapid deterioration and a high mortality rate. It may lead to functional disorders of the lungs, liver, kidneys, and other organs, severely compromising the life safety of patients [12]. ARDS is characterized by pulmonary edema due to alveolar inflammatory exudate and increased pulmonary vascular permeability, which leads to impaired gas exchange and acute deterioration, and its mechanism is still poorly understood [13]. In patients with ARDS, early and effective pharmacotherapeutic interventions to reduce ventilator dependence are essential for the enhancement of patients' survival. In this study, budesonide/glycopyrronium bromide/formoterol (Breztri Aerosphere) were adopted for the treatment of ARDS patients and have achieved promising results.

Herein, Breztri Aerosphere achieved a higher total efficacy (93.33% vs. 76.67%), significantly lower APACHE II scores and Murray lung injury scores, and higher levels of PCO_2_, PO_2_, and SaO_2_ versus conventional treatment. Budesonide/glycopyrronium bromide/formoterol (Breztri Aerosphere) is a fixed-dose triple inhalation formulation that uses an innovative co-suspension delivery technology to deliver budesonide (inhaled glucocorticoid)/glycopyrronium bromide (long-acting anticholinergic)/formoterol fumarate (long-acting *β*2 agonist). Analysis of positive results of the phase III ETHOS trial showed that in patients with moderate to very severe COPD, the rate of moderate to severe acute exacerbations was reduced by 24% and 13% after the use of budesonide/glycopyrronium bromide/formoterol (Breztri Aerosphere) compared to the dual therapy of glycopyrronium bromide/formoterol fumarate and budesonide/formoterol fumarate [14]. Anti-inflammatory drug therapy is considered the bedrock of ARDS pharmacotherapy. In the early stage of ARDS, an immune reaction in the body in response to local or systemic injury may be associated with the release of inflammatory cells and inflammatory mediators in the lungs, which underscores the significance of regulating the proinflammatory system. Glucocorticoids are currently the most frequently used drugs to inhibit the inflammatory response in clinical practice, which can promote the secretion of alveolar surface-active substances from the alveolar type II epithelial cells, maintain cellular stability, reduce microvascular permeability, and promote pulmonary edema absorption, thus driving down the release of inflammatory mediators and minimizing cellular damage. Moreover, they can also inhibit fibroblast proliferation and collagen deposition and hamper the progression of pulmonary fibrosis [15]. In this study, Breztri Aerosphere obtained a significantly higher SVR level and significantly lower levels of PVR, MAPA, and PAWP versus conventional treatment, which is consistent with the research results of a previous study which pointed out that the administration of moderate doses of glucocorticoids in the early stages of ARDS may contribute to improving oxygenation on the 28th day after onset, enhancing pulmonary function, and avoiding infections and the occurrence of infectious shock in patients with ARDS [16]. The results of this study demonstrated that after treatment, the levels of IL-6, IL-10, TNF-*α*, and PCT decreased significantly in both groups, with lower results seen in patients receiving Breztri Aerosphere. It has been confirmed that one of the etiologies of ARDS lies in the acute impairment of pulmonary microcirculatory function due to the massive release of acetylcholine, high vagal excitation, sustained pulmonary microvascular spasm, and increased pulmonary capillary permeability in the body [17]. Research has illustrated that anticholinergic drugs are effective in the suppression of the activation of effector cells such as neutrophils, the reduction of inflammatory factor release, and the mitigation of acute lung injury [18]. In addition, *β*2 agonists are extensively used in the treatment of asthma and COPD and serve to block several pathogenic aspects of ARDS, restore or improve the permeability of pulmonary microvascular endothelium and alveolar epithelium, inhibit the release of inflammatory mediators, regulate the activity and secretion of alveolar surface-active substances, and enhance Na^+^-K^+^-ATP enzyme activity, which is consistent with the results of the present study [19].

RETRACTED

## 5. Conclusion

Adjuvant therapy with budesonide/glycopyrronium bromide/formoterol (Breztri Aerosphere) in ARDS patients can significantly reduce APACHE II scores and Murray lung injury scores, improve blood gas indexes and pulmonary circulation function indexes, and shorten mechanical ventilation time and ICU time, which may be attributed to its improvement of organism inflammation status and reduction of inflammatory factors.

## Figures and Tables

**Figure 1:** Comparison of APACHE II scores and Murray lung injury scores between the two groups of patients. Note: ^*∗∗∗*^*P* < 0.001.

**Figure 2:** Comparison of SVR, PVR, MAPA, and PAWP between the two groups of patients. Note: ^*∗∗*^*P* < 0.01; ^*∗∗∗*^*P* < 0.001.

**Figure 3:** Comparison of the serum levels of IL-10, TNF-*α*, and PCT between the two groups of patients. Note: ^*∗∗*^*P* < 0.01; ^*∗∗∗*^*P* < 0.001.

**Figure 4:** Comparison of the survival curve between the two groups of patients.

**Table 1:** Comparison of general information between the two groups of patients.

	Control group (*n* = 60)	Study group (*n* = 60)	*χ*2/*t*	*P*
Age (years)	62.35 ± 12.23	60.46 ± 14.35	0.777	0.439
Gender (male/female)	41/19	38/22	2.580	0.108
BMI (kg/m^2^)	26.45 ± 5.31	25.97 ± 6.43	0.446	0.657
Primary illness			1.006	0.800
Pulmonary infection	36	38		
Extrapulmonary infection	14	10		
Shock	6	8		
Others	4	4		

**Table 2:** Comparison of clinical efficacy between the two groups of patients.

	Cured	Effective	Ineffective	Total effective rate
Control group (*n* = 60)	12	34	14	46
Study group (*n* = 60)	16	38	6	54
*χ* ^2^				6.539
*P*				0.011

**Table 3:** Comparison of blood gas indexes between the two groups of patients.

	PCO_2_ (mmHg)		PO_2_ (mmHg)		SaO_2_ (%)	
	Before	After	Before	After	Before	After
Control group (*n* = 60)	50.24 ± 8.34	56.34 ± 6.77	69.24 ± 8.24	76.23 ± 9.23	82.34 ± 4.45	90.35 ± 6.31
Study group (*n* = 60)	48.93 ± 9.34	61.28 ± 7.03	70.29 ± 7.23	82.34 ± 6.23	81.94 ± 5.02	93.45 ± 6.26
*t*	0.810	3.921	0.742	4.250	0.462	2.702
*P*	0.419	<0.001	0.460	<0.001	0.645	0.008

RETRACTED

**Table 4:** Comparison of mechanical ventilation time and ICU time between the two groups of patients.

	Cases of mechanical ventilation	Mechanical ventilation time	ICU time
Control group (*n* = 60)	52	5.27 ± 1.58	6.58 ± 2.04
Study group (*n* = 60)	49	4.16 ± 1.24	5.47 ± 1.79
*χ* ^2^/*t*	0.563	3.912	3.168
*P*	0.453	<0.001	0.002

## Data Availability

The datasets used during the present study are available from the corresponding author upon reasonable request.
